The article "Tap versus Bottled Water in Kampala, Uganda: Analyses of Consumers' Perception alongside Bacteriological and Physicochemical Quality" was published in 2022. Journal: J Environ Public Health.

# Tap versus Bottled Water in Kampala, Uganda: Analyses of Consumers' Perception alongside Bacteriological and Physicochemical Quality

**DOI:** 10.1155/2022/9336247

**Published:** 2022-04-25

**Authors:** Charles Onyutha, Josephine Taata Akobo, Ambrose Mubialiwo

**Affiliations:** Department of Civil and Environmental Engineering, Kyambogo University, P.O. Box 1, Kyambogo, Kampala, Uganda

## Abstract

In Uganda, tap water is always ensured to be potable. However, people are not sure whether tap water is generally safe for drinking without being boiled. Conversely, bottled water consumption is on the increase in Uganda. The main problem lies in the cost of energy for boiling tap water or purchasing bottled water. This study analyzed results of laboratory tests and consumers' perception for comparison of tap and bottled water in Nakawa division, Kampala. Tap water was sampled at four representative locations. At least 16 different brands of bottled water were considered. The top four most consumer-preferred bottled water brands were selected for further analysis. In our study, 28.8%, 6.06%, and 13.64% of the 142 respondents indicated that bottled water had taste, color, and smell, respectively. However, 27.5%, 25.4%, and 34.5% of the respondents agreed that tap water had taste, color, and smell, respectively. Both tap and bottled water met the World Health Organization (WHO) guidelines for pH, total dissolved solids, chloride, copper, sodium, sulfate, and nitrate. However, a tap water sample was found to contain Coliform bacteria. In this line, affected communities need to thoroughly boil the raw tap water to kill the pathogens. All tap water samples yielded iron concentrations above the WHO recommended limit. Student's *t*-tests showed that tap and bottled water samples were significantly (*p*<0.05) different with respect to total dissolved solids, pH, chloride, calcium, magnesium, iron, sodium, sulfate, and nitrate. We emphasize the need for routine maintenance of the water distribution system to check for leakages which can be potential source of contaminations.

## 1. Introduction

Up to 60% of a human body comprises water. Thus, it is commonly believed that water is life. Safe drinking water, human health, and well-being are interlinked; see, for example, [1] and World Health Organization [2, 3]. In the same line, Target 6 of the United Nations Sustainable Development Goals aims at ensuring availability and sustainable management of water and sanitation for all [4]. In a relevant development, the Government of Uganda (GoU) established the Uganda Vision 2040 framework in 2013 to improve the health, sanitation, and hygiene, as well as promoting commercial and low consumption industrial arrangements [5]. Eventually, the National Water and Sewerage Corporation (NWSC), a utility parastatal solely owned by the GoU, is committed to providing clean and safe water in almost all towns and urban centers across Uganda. The overall potable water service coverage by 2020 was at 74% (Ministry of Water and Environment MWE [6]) despite the NWSC's commitment in reaching the milestone of 100%. The extension of piped water supply system takes into consideration the urbanization strategy which the GoU is promoting over the Vision 2040 period. The NWSC's customer satisfaction index was 88% for the year 2015/16 but dropped to 77% in 2019/20 [6]. Water supply systems in urban areas need constant monitoring and repairs of leakage points to guide against pathogen intrusion which can contaminate the drinking water. In Kampala (the capital city of Uganda), the biggest percentage (about 76.7%) of the total community population in slums get their water from piped water system, and most (or 97.2%) of these people understand the danger related with consuming unsafe water, and they eventually boil water for drinking [7]. Taking raw or unboiled water can lead to waterborne diseases such as cholera, dysentery, and typhoid. For instance, Kampala City Council Authority (KCCA) alerted the Ugandan Ministry of Health of a “strange disease” that killed one person and sickened dozens in 2015. In a follow-up study by Kabwama and others [8] from 17 February to 12 June 2015, the strange disease was related to consumption of water and drinks contaminated by feces. In 2018, an outbreak of cholera (a waterborne disease) in Kampala was declared by Ministry of Health with seven confirmed cases [9].

Currently, the issues of tap water have made it very challenging to persuade communities especially in urban centers and neighboring slums to consume tap water as most of them are changing to the use of bottled water [10]. Like in other places across the world, bottled water has become a very common consumer product in the various towns and cities of Uganda. On average, a 500 ml or 650 ml bottled water costs between Uganda Shillings (UGx) 1000 and 1,500 UGx (or 0.27 and 0.41 US$) while a 20-litre jerrycan of tap water costs about 300 UGx (or 0.08 US$). Considering only the brands certified by the Uganda National Bureau of Standards, there are about 100 bottled water brands available in market. Differences in brands occur with respect to cost, bottle capacity, taste, color, and odor among others. These differences influence the choice of which bottled water one can consume.

Whether one needs to drink tap or bottled water, the quality of the drinking water needs to always be ascertained. To assess the quality of water consumed in Uganda, several studies [7, 11–14] have been conducted. These previous studies had a number of research gaps. For instance, none of the cited studies undertook comparison of both tap and bottled water. Besides, the past studies did not consider the component of initial market survey to obtain the most consumer-preferred and common brands available in the market. Some studies like Ssemugabo and others [7] lacked analysis of laboratory tests of water samples. Nevertheless, the quality of both tap and bottled water should always be updated at a given location as part of the required practices for assessment and surveillance of drinking water quality. Therefore, this study aimed at comparing tap and bottled water while analyzing consumers' perception and water quality laboratory test results.

## 2. Materials and Methods

### 2.1. Study Area

Banda parish located in Nakawa division of the KCCA (Figure 1) was selected as the study area. By 2014, about 5% of the total households in Nakawa never had access to safe water [15]. Banda is one of the slums in Kampala. Banda parish comprises a total of eleven zones (Zone B1 to B11). Banda has about 10,000 households, with a total population of nearly 50,000 [16]. The parish has key landmarks such as Kyambogo University, Mogas Petroleum tanks, Banda community, Nabisunsa Girls Secondary School, Kyambogo College School, a number of fuel filling stations (also called Petrol stations), and the Ministry of Works and Transport Laboratory. The parish covers a total land area of about 0.6 km^2^ (150 acres). Springs, boreholes, wells, piped water, and bottled water are the available sources of drinking water in the study area. Malaria and waterborne diseases such as cholera, diarrhea, and typhoid are some of the leading causes of morbidity and mortality in Banda parish. Just like in the various parts of Uganda, Banda parish has several bottled water brands available in the market.

### 2.2. Data Collection and Analysis

#### 2.2.1. Research Design and Assessment of the Available Bottled Water Brands

This study employed experimental and ethnographical designs. Using a survey sheet, different bottled water brands available in each shop and/or supermarket were identified. A questionnaire was also given to the locals or inhabitants of the study area to determine (i) which bottled water brands were preferred to others (here, a total of 311 consumers participated) and (ii) community perception regarding taste, color, and smell of both tap and bottled water (and this was based on a sample of 142 consumers). Possible differences in perception due to the possible influence of gender on water quality taste, color, and smell were investigated.

Tap water was sampled from a total of four zones which were considered representative of the study area (or Banda parish). Unflushed tap water was sampled at four locations between 9 : 00 am and 10 : 30 am on the November 5, 2020. At each location, water was sampled using clean plastic bottles of capacity 500 ml from nonmixing (only cold water) faucets in the kitchen sinks. The water from the kitchen sinks was considered to be fresh since it comes directly from the water supply distribution main. Water from the storage tanks was avoided to eliminate influence from possible cases of contamination of the water to be sampled due to storage issues stemming from poor maintenance of the water tanks. The researcher collecting the water sampled wore clean and new gloves. During sampling process, the lid of each water sampling bottle was carefully opened and put in position to receive the tap water. The faucet was opened and the 500 ml sampling bottle was filled with the tap water. The samples were placed in a clean container with a lid. The samples were then transported by a car to the Uganda Industrial Research Institute (UIRI) laboratory where the water quality tests were conducted. UIRI laboratory was selected because it is certified by the Uganda National Bureau of Standards, and it is very near to the tap water sampling locations. From the time of collecting the last sample, it took less than 20 minutes for transporting the samples to the laboratory.

Samples from the top four consumer-preferred bottled water brands were also taken to the laboratory for water quality tests. The sampling comprised buying a bottle of each of the four bottled water brands from a shop, placing the bottled water in a clean box and transporting them to the UIRI laboratory. Each bottled water was ensured to have its date of purchase far from the expiry date. The choices of the top four consumer-preferred brands and four representative tap water sampling zones were to permit a number of laboratory tests to be conducted for ascertaining both bacteriological and physicochemical properties of the drinking water. The tests conducted on each water sample included pH, total dissolved solids (TDS), chloride, calcium, magnesium, copper, iron, sodium, sulfate, nitrate, and*Escherichia coli*. The results obtained were compared with the drinking water standards based on the WHO [3] guidelines. Brief descriptions of the laboratory tests are given in Appendix A.

#### 2.2.2. Analysis of the Difference between Tap and Bottled Water

To evaluate the difference between tap and bottled water with respect to a number of water quality parameters, a null hypothesis *H*_0_ (the mean of a parameter like pH from tap water ${\bar{x}}_{1}$ was the same as that from bottled water ${\bar{x}}_{2}$) was analyzed. To test such a hypothesis, we use Student's *t*-test and z-test when the sample size is less (or equal to) and greater than 30, respectively. In this study, Student's *t-test* [17] statistic was computed using

(1) $$\begin{array}{c} t=\left({\bar{x}}_{i}-{\bar{x}}_{2}\right)\times {\left(s_{s}\sqrt{\frac{1}{n_{1}}+\frac{1}{n_{2}}}\right)}^{-1}, \end{array}$$

and

(2) $$\begin{array}{c} s_{s}=\sqrt{\frac{\left(n_{1}-1\right)s_{1}{}^{2}+\left(n_{2}-1\right)s_{2}^{2}}{n_{1}+n_{2}-2}}, \end{array}$$

where *s*_1_ and *s*_2_ denote the standard deviations of the parameters (such as pH) from the tap and bottled water samples, respectively. In the same line, ${\bar{x}}_{1}$ and ${\bar{x}}_{2}$ are the mean values of the parameters (such as pH) from the tap and bottled water samples, respectively. Lastly, *n*_1_ and *n*_2_ denote the sample sizes of tap and bottled water samples, respectively. Sample size determines degree of freedom in the *t*-test. As the sample size increases, the tail of the Student's *t*-distribution gets thinner. However, the tail of the *t*-distribution is thick when the sample size is small. The thickness or thinness of the tail of the Student's *t*-distribution can affect the rejection rates for the *H*_0_. The *H*_0_, $\left({\bar{x}}_{1}={\bar{x}}_{2}\right)$ was rejected for *p* value less than *α* = 0.05; else, the *H*_*o*_ was not rejected.

## 3. Results and Discussion

### 3.1. Available Bottled Water Brands in the Market

Table 1 shows the preference of bottled water brands by the respondents. The brands were allocated arbitrary numbers 1 to 16 (not exact names to avoid bias during the survey). Brands 1, 3, 2, and 5 were the most consumed bottled water brands with overall consumption percentages of 52.1, 21.5, 8.7, and 4.5% of the respondents, respectively (Table 1). Brand 13 had the least percentage (0.3%). Whereas 16 bottled water brands had been consumed at least once by each respondent, seven of them (brands 4, 6, 9, 11, 12, 13, and 16) were not available in the sampled shop outlets and/or supermarkets in the study area (Table 2). Thus, the quality parameters for these brands are missing in Table 2. The percentages of males and females for each of the top four bottled water brands were comparable or not significantly different (*p* = 0.3916 or *p* > 0.05). Furthermore, a linear relationship between the data from males and females yielded coefficient of determination *R*^2^ of 0.989. This meant that the variance in the choices of the males could adequately be explained using those of females. Thus, the consumer's choice of the bottled water brands was not linked to gender.

### 3.2. Consumer Perception on Water Quality in terms of Taste, Odor, and Color

Taste and odor in water may be produced by either organic or inorganic materials. The perceptions of taste and odor are closely related and often confused by both water practitioners and consumers. Generally, a substance that produces odor in water almost invariably imparts a perception of taste as well [18, 19]. Objectionable concentration may depend on social and cultural factors. Pure water should ideally be colorless. However, foreign substances such as organic matter from soils, vegetation, minerals, and aquatic organisms present in water tend to give water some color. Color can also be contributed by municipal and industrial wastes [19]. Color above 15 true color units (TCU) can be detected by humans in a glass of water [3].

Figure 2 shows the consumer perception on the quality of tap and bottled water in terms of taste, odor, and color, respectively. From Figures 2(b) and 2(e), about 28.78% of the sampled consumers suggested that bottled water had taste, while 62.88% disagreed with the statement “bottled water has taste.” Regarding tap water, 27.47% of the consumers suggested that tap water had taste, while 61.27% of the respondents disagreed with the statement “tap water has taste.” The mean of consumers' response or perception on bottled water was 26.4 ± 18.13 while that on tap water was 28.4 ± 14.11. A higher variability was observed in the perception on bottled water (standard deviation or Stdev = 18.13) than tap water (Stdev = 14.11). However, it is clear that almost the same percentage agreed and/disagreed with the statements on the taste on both tap and bottled water.

Regarding the perception on odor in Figures 2(c) and 2(f), only 13.64% of the sampled consumers suggested that bottled water had smell, while a large percentage (80.3%) of the respondents objected the statement “bottled water has smell.” On the other hand, 34.51% acknowledged that tap water had smell, while 58.45% disagreed with the statement “tap water has smell.” From these values, it is clear that tap water was more highly considered to have smell than bottled water. This could be one of the reasons for the increasing demand of bottled water. The mean value for the consumers' responses on smell in bottled water was 26.4 ± 31.8. For tap water, the mean ± Stdev of the responses was 28.4 ± 13.7. Similar to taste, responses on bottled water in terms of smell exhibited higher variability (Stdev = 31.8) than those on tap water (Stdev = 13.7).

Community perception on color Figures 2(a) and 2(d) showed that 87.88% of the sampled consumers regarded bottled water to have no color while 6.06% of the respondents stated that bottled water had color. The mean of response and standard value of the perception on color in bottled water were 26.4 and 34.2, respectively. On the other hand, 25.35% of the respondents regarded tap water to have color while majority (71.13%) of the sampled consumers disagreed with the statement “tap water has color.” The mean ± Stdev of consumers' responses on color of tap water was 28.4 ± 20.9. Similarly, from the above values, it is noticeable that tap water was more highly considered to have color than bottled water. This could as well be one of the reasons for the increasing demand of bottled water. As previously observed with taste and smell, the perception on bottled water in terms of color showed the higher variability (Stdev = 34.2) than on tap water (Stdev = 20.9).

The proportions of the males and females in the sampled consumers were 37.12 and 62.88%, respectively (Figures 2(a)–2(f)). In other words, females were larger in number than males. Our findings are consistent the the results of another study [11] which was conducted for the same study area and indicated that the proportions of males and females sampled to determine perception of consumers regarding local water treatment were 36% and 64%, respectively. The study conducted by Qian [10] in three regions of Singapore, Hong Kong, and Macau also reported higher percentages of females than male. This could be attributed to the fact that females interact more with water especially in doing domestics chores than men, hence giving females more information about the water qualities. For instance, 80% of the persons responsible for fetching water in the study area comprise women compared with children (15%) and men (05%) [11].

### 3.3. Comparative Analysis of Tap and Bottled Water

Samples from bottled water brands 1, 2, 3, and 5 were labeled as BW1, BW2, BW3, and BW4, respectively. TW1, TW2, TW3, and TW4 represent samples of tap water from Banda, zones B3, B7, B10, and B11, respectively. Results of laboratory tests plotted in Figure 3 are also summarized in Table 3. The dotted and dashed horizontal lines in Figures 3(a)–3(h) show the limits from the WHO [3] water quality guidelines. The WHO [3] directive parametric values of pH, TDS, chloride, copper, iron, sodium, sulfate, and nitrate are 6.5–8.5, 1000 mg/L, 250 mg/L, 2 mg/L, 0.2 mg/L, 200 mg/L, 250 mg/L, and 50 mg/L, respectively. Parametric values for calcium and magnesium were not given. According to WHO [3], *Escherichia coli* or E.*coli* (cfu/100 ml) should be absent in a drinking water sample.

Presence of high levels of TDS in water may be unpleasant to consumers because of the resulting taste and undue scaling in water pipes, heaters, boilers, and household appliances. Water with extremely low concentrations of TDS may also be intolerable to consumers because of its flat, dull taste and corrosiveness to water-supply systems [19].  Figure 3(a) shows TDS of tap and bottled water. Both tap and bottled water had the TDS lower than the limit of 1000 mg/L. The TDS of tap water in mg/L ranged from 100 to 104.6 while that of bottled water varied from 16.7 to 90.6. The TDS of tap water had mean ± Stdev of 102.1 ± 2.1 mg/L, while that of bottled water was 54.8 ± 34.61 mg/L. The difference between the means of TDS from tap and bottled water was significant (*p* = 0.031 or *p* < 0.05).

Samples obtained from tap water showed pH above 7 (basic conditions). The pH of bottled water was slightly below that of tap water (Figure 3(b)). However, both tap and bottled water in the study area met the pH requirements. The pH of tap and bottled water had mean ± Stdev of 8.06 ± 0.15 and 7.0 ± 0.063, respectively. However, the difference between the means of pH from tap and bottled water was significant (*p* = 0.0001 or *p* < 0.05). The pH of bottled water was closer to 7 than that of tap water (Figure 3(b)). Generally, water with a pH < 7 is considered acidic and one with a pH > 7 is regarded alkaline. Water with a pH > 8.5 denotes hard water. Long-term consumption of hardwater may lead to kidney dysfunction which may result in further complicated diseases such as diabetes [20].

Both tap and bottled water were found to have quantities of sulfate way less than the maximum parametric value 250 mg/L (Figure 3(c)). Sulfate has an effect on taste. Taste impairment varies with the nature of the associated cation. The taste thresholds have been found to range from 250 mg/L for sodium sulfate to 1000 mg/L for calcium sulfate. Therefore, the sulfate present in the water sampled from the study area was deemed to have no effect on the taste of water given that it was below the maximum parametric limit. Sulfates in tap and bottled water exhibited mean ± Stdev of 16.7 ± 1.56 mg/L and 4.18 ± 2.4 mg/L, respectively. The difference between the means of sulfates from tap and bottled water was significant (*p* = 0.0005 or *p* < 0.05). Sulfates are found in almost all-natural waters, and the concentration varies according to the nature of the terrain through which they flow. Sulfates are discharged into water via industrial wastes and through atmospheric deposition. They are often derived from the sulfides of heavy metals such as iron, copper, and lead. Sulfate when combined with calcium and magnesium makes water hard.

Nitrate concentrations in both tap and bottled water were below the recommended maximum value of 50 mg/L (Figure 3(d)). The amount of nitrate in bottled water ranged from 1.1 to 4.6 mg/L, while that of tap water varied over range 10.7–16.7 mg/L. Tap water had nitrate content higher than that of bottled water. The nitrate amounts found in tap water exhibited mean ± Stdev of 14.2 ± 3.0 mg/L while that in bottled water was 3.1 ± 1.62 mg/L. There was a significant (*p* = 0.0016 or *p* < 0.05) difference between the means of the nitrate amounts from tap and bottled water. Nitrate is found naturally in the environment. Nitrate and nitrite can be ingested in water when free ammonia enters the water in the water distribution system. High nitrate levels are often associated with increased microbiological contamination. This is because nitrates can emanate from sewage.

Both tap and bottled had the chloride values less than the WHO [3] directive parametric stipulation of 250 mg/L (Figure 3(e)). Chloride values in bottled water ranged from 3.8 to 6.1 mg/L and were less than the values from tap water (29.5–44.1 mg/L). Chlorides in drinking water do not lead to any harmful effects on public health, but high concentrations can lead to a salty taste which makes most people find objectionable. When chlorides are present in concentrations more than 250 mg/L, the taste of the water may be unpleasant to some consumers. However, some consumers can become accustomed to low levels of chloride-induced taste. Taste thresholds for the chloride anion depend on the associated cation and are in the range of 200–300 mg/L for sodium, potassium, and calcium chloride. The total chloride in tap water had mean ± Stdev of 36.1 ± 6.24 mg/L while that of bottled water was 5.02 ± 1.15 mg/L. The difference between the free chlorine in tap and bottled water samples was significant (*p* = 0.0003 or *p* < 0.05). No health-based guideline value is proposed for chloride in drinking water. Chloride concentrations found in drinking water from the study area may not be of serious health concern though they may affect acceptability of drinking water [3].

The amounts of copper in both tap and bottled water were lower than the maximum recommended value of 2 mg/L (Figure 3(f)). However, the amounts of copper in tap water (0.12–1.17 mg/L) were larger than those in bottled water (0.001–0.003 mg/L). The total copper ions in tap and bottled water had mean ± Stdev of 0.62 ± 0.56 mg/L and 0.002 ± 0.001 mg/L, respectively. The difference in the means of copper concentration in tap and bottled water was insignificant (*p* = 0.053 or *p* > 0.05). Copper is found in some natural waters, particularly in areas where ore deposits have been mined. In drinking water, copper can occur in corrosive water that passes through copper pipes. Copper concentrations in treated water often increase during distribution, especially in systems with an acidic pH or high-carbonate waters with an alkaline pH. Presence of large copper concentration in drinking water may negatively affect human health. However, copper in small amounts has no effect on health, but will impart an undesirable taste to the drinking water [21].

Bottled water was found to have iron concentrations much less than the WHO parametric value 0.2 mg/L while all samples of tap water had iron concentrations far greater than 0.2 mg/L (Figure 3(g)). Drinking water with iron has health benefits. However, high concentrations of iron may negatively impact human health. Besides, presence of iron in water is considered objectionable because it imparts a brownish color in the water and affects the taste of water [21]. There is usually no noticeable taste at iron concentrations below 0.3 mg/L. No health-based guideline value is proposed for iron. The total iron concentrations in tap and bottled water had mean ± Stdev of 1.65 ± 0.81 mg/L and 0.023 ± 0.015 mg/L, respectively. The difference between the means of iron concentrations in tap and bottled water was significant (*p* = 0.0088 or *p* < 0.05). Iron can be naturally found in groundwater and some surface water (such as creeks, rivers, and certain shallow dug wells). Drinking water may pick up iron as it flows through rusty steel or cast-iron pipes [21]. Iron comes in either dissolved or suspended form. Exposure of dissolved iron to air makes the water turn to black or orange.

Both tap and bottled water yielded sodium concentrations below the WHO [3] parametric value of 200 mg/L for sodium (Figure 3(h)). Sodium concentrations in tap and bottled water were in the ranges 17.6–22.6 mg/L and 5.5–11.1 mg/L, respectively. Sodium concentrations in tap and bottled water had mean ± Stdev of 19.9 ± 2.1 mg/L and 8.35 ± 2.7 mg/L, respectively. The difference between the means of sodium concentrations in tap and bottled water was found to be significant (*p* = 0.0015 or *p* < 0.05). Sodium occurs naturally in the Earth's crust and may not be considered toxic. The taste threshold concentration of sodium in drinking water depends on the anion present as well as the temperature of the water. Sodium salts are found in virtually all food (the main source of exposure) and drinking water. High sodium intake has partially been proven to increase risk of hypertension [22]. It still remains unknown whether the consumption of sodium in drinking water could have similar effects on health [22]. No health-based guideline value has been derived as the daily contribution of sodium from drinking water is small.

Directive parametric value for calcium was not stipulated in the WHO [3]. Nevertheless, the taste threshold for the calcium ion is in the range of 100–300 mg/L depending on the associated anion [23]. In this study, tap and bottled water yielded calcium concentrations below the taste threshold for calcium ion in water (Figure 3(i)). Tap water was found to have higher values of calcium (ranging from 55.3 to 73 mg/L) than bottled water (1.99–9.8 mg/L). The total calcium in tap water had mean ± Stdev of 66.65 ± 7.8 mg/L and 6.9 ± 3.4 mg/L, respectively. The difference between the means of calcium concentrations in tap and bottled water was significant (*p* = 0.0001 or *p* < 0.05). Calcium ions and salts are very common in water, and in most natural fresh water, calcium is the principal cation. It is also the most abundant element in the human body and its intake is essential for normal growth and health including drop of pregnancy hypertensive disorders and lowers blood pressure mainly among young individuals [24]. Calcium is useful in the strengthening of bones and teeth. The maximum daily requirement is of the order 1–2 grams and comes in the form of dairy products. However, excessive consumption of water with high concentration of calcium may lead to the formation of concretion in the organs such as kidneys or urinary bladder and may give rise to irritation of the urinary passages resulting in difficulties in passing urine. Hardness of water can cause wastage of soap and scale formation.

Like for calcium, parametric value for magnesium concentration was not stipulated by the WHO [3]. Tap water was found to have higher values of magnesium (fluctuating between 23.9 and 37.8 mg/L) than those of bottled water (varying from 0.42 to 3.9 mg/L) (Figure 3(j)). The total magnesium in tap and bottled water had mean ± Stdev of 32.2 ± 6.4 mg/L and 2.5 ± 1.6 mg/L, respectively. The difference between the means of magnesium concentrations in tap and bottled water was significant (*p* = 0.0005 or *p* < 0.05). The presence of magnesium in drinking water has far reaching benefits including prevention of million heart disease and stroke deaths annually [25]. Besides, magnesium is second to calcium in causing water hardness.

Results on Coliform bacteria are shown in Figure 4. Coliform bacteria were only found in TW2 or tap water sampled in zone B7 Banda. Total coliform bacteria (excluding *E. coli*) occur in both sewage and natural waters. Coliforms are heterotrophic and able to multiply in water and soil environments. Total coliforms include organisms that can survive and grow in water. They can be used to assess the cleanliness and integrity of distribution systems and the potential presence of biofilms. The presence of coliform bacteria in water is an indicator for fecal contamination. Since they can survive and multiply in plant material, soil, sediments in water reservoirs, they also indicate the intrusion of soil into drinking-water reservoirs. However, total coliforms are less suitable as indicator organisms [3].

Generally, *E. coli* in both tap and bottled water in cfu/100 ml was less than one. Blue colonies indicate the presence of *E. coli*. In this study, there was no presence of *E. coli* in both tap and bottled water. *E. coli* are typically excreted in the feces of humans and other warm-blooded animals. Most *E. coli* strains are nonpathogenic and reside harmlessly in the colon. However, certain serotypes (such as *E. coli* O157 : H7) do play a role in intestinal and extra-intestinal diseases, such as urinary tract infections, and have been involved in drinking-waterborne outbreaks. *E. coli* is the most widely used indicator of fecal pollution in water. Detection of *E. coli* should lead to further action, like additional sampling and investigation of potential sources such as inadequate treatment or breaches in distribution system integrity. *E. coli* should be checked in any water to ascertain quality since it is a bacteria indicator which works as an early sentinel of possible health hazards for the community [26].

## 4. Conclusion

This study conducted market survey to determine the most commonly available bottled water brands in Banda, a slum of Kampala (or the capital city of Uganda). A total of 311 consumers were interviewed on which bottled water brands they liked most. Through questionnaire, perceptions of a total of 145 consumers regarding taste, smell and color of both tap and bottled water were assessed.

The top four bottled water brands which the consumers liked obtained 52.1, 21.5, 8.7, and 4.5% of the responses, respectively. A total of 28.78, 6.06, and 13.64% of the consumers agreed that bottled water had taste, color, and smell, respectively. On the other hand, 27.47, 25.35, and 34.5% of the consumers agreed that tap water had taste, color, and smell, respectively. Both tap and bottled water met the WHO [3] directive parametric values for pH, TDS, chloride, copper, sodium, sulfate, and nitrate. The differences between the mean values of test results for tap and bottled water were found to be significant (*p* < 0.05) with respect to pH, TDS, chloride, calcium, magnesium, iron, sodium, sulfate, and nitrate. However, the difference between the means of copper concentrations in tap and bottled water samples was insignificant (*p* > 0.05). Both tap and bottled water generally did not contain *E. coli*. Only one tap water sample (TW2) contained Coliform bacteria. The contamination in tap water could be due to fecal contamination, or soil intrusion during water distribution, rusty steel pipes or cast-iron pipes. In such a case, affected communities can continue with the culture of boiling water to kill possible pathogens which may be present in the distributed water. Boiling tap water can make the consumers to be sure about the quality of the water they have to drink. Importantly, there is need for routine maintenance of the distribution system to check for leakages which can be potential source of contaminations.

As part of the required practices for assessment and surveillance of drinking water quality, future research to be conducted in the various slums in Uganda need to take into account (i) the effect of seasonality on quality of tap water given the sustained performance of water treatment plants, (ii) deterioration of bottled water brands in market due to storage and handling, (iii) the factors influencing the community choice for bottled water as a replacement for tap water, and (iv) the difference in the cost of boiling tap water and refining the tap water quality through chemical or biological treatment means.

## Figures and Tables

**Figure 1:** The study area adopted from [11].

**Figure 2:** Consumers' perception on the (a, d) taste, (b, e) color, and (c, f) smell of (a, b, c) tap water and (d, e, f) bottled water.

**Figure 3:** Comparison of tap and bottled water with respect to (a) TDS, (b) pH, (c) sulfate, (d) nitrate, (e) chloride, (f) copper, (g) iron, (h) sodium, (i) calcium, and (j) magnesium.

**Figure 4:** Presence of Coliform bacteria in (a) TW1 and (b) TW2.

**Table 1:** Bottled water brands consumed by the respondents.

Water brand	Males		Females		Total	
	Number	Percentage	Number	Percentage	Number	Percentage
1	88	55.3	74	48.7	162	52.1
2	12	7.5	15	9.9	27	8.7
3	33	20.8	34	22.4	67	21.5
4	1	0.6	1	0.7	2	0.6
5	7	4.4	7	4.6	14	4.5
6	0	0.0	1	0.7	1	0.3
7	5	3.1	3	2.0	8	2.6
8	2	1.3	4	2.6	6	1.9
9	2	1.3	4	2.6	6	1.9
10	1	0.6	1	0.7	2	0.6
11	2	1.3	1	0.7	3	1
12	2	1.3	3	2.0	5	1.6
13	0	0.0	1	0.7	1	0.3
14	2	1.3	1	0.7	3	1
15	1	0.6	1	0.7	2	0.6
16	1	0.6	1	0.7	2	0.6
Total	159	100	152	100	311	100

**Table 2:** Water quality parameters indicated on the bottle of each brand.

Water brand	Water quality parameters										
	Fe	K	Ca	NO_3_^2−^	Na	F	Cl	Mg	Cu	TDS	SO_3_^2−^
1	P	P	P	P	P	P	P	P		P	P
2	P	P	P		P	P	P	P			
3	P	P	P	P	P	P	P	P	P	P	
4											
5	P	P	P		P	P	P	P	P		
6											
7	P	P	P		P	P	P	P		P	P
8	P	P	P		P	P	P	P		P	P
9											
10	P	P	P		P	P	P	P		P	P
11											
12											
13											
14	P	P			P	P	P				
15	P	P	P	P		P	P	P	P		
16											

The blank parts indicate absent while P denotes present.

**Table 3:** Results of water quality laboratory tests.

Sample	BW1	BW2	BW3	BW4	TW1	TW2	TW3	TW4
pH	6.94	6.84	7.01	7.02	7.85	8.07	8.17	8.16
TDS (mg/L)	90.6	16.7	76.7	35.3	100	100.8	104.6	102.8
Chloride (mg/L)	6.1	4.3	5.9	3.8	33.4	44.1	37.5	29.5
Calcium (mg/L)	9.8	1.99	7.3	8.4	70.2	73	55.3	68.1
Magnesium (mg/L)	3.9	0.42	2.24	3.5	36.5	37.8	23.9	30.5
Copper (mg/L)	0.003	0.001	0.001	0.002	0.12	0.16	1.17	1.02
Iron (mg/L)	0.04	0.01	0.03	0.01	1.04	0.88	2.43	2.26
Sodium (mg/L)	10.2	5.5	11.1	6.6	20.2	17.6	22.6	19
Sulfate (mg/L)	3.8	1.6	7.4	3.9	18.1	15.9	14.9	17.9
Nitrate (mg/L)	4.6	1.1	4.2	2.5	12.7	10.7	16.7	16.7
*Escherichia coli* (cfu/100 ml)	<1	<1	<1	<1	<1	<1	<1	<1

**Table 4:** References for water quality tests.

S. no.	Test	Reference
1	Determination of pH	ISO 10523
2	Determination of sulfates	ISO 22743
3	Determination of the sum of calcium and magnesium	ISO 6059
4	Determination of the chemical oxygen demand	ISO 6332
5	Determination of nitrate	ISO 7890
6	Determination of calcium and magnesium	ISO 7980
7	Determination of iron	ISO 6332
8	Determination of cobalt, nickel, copper, zinc, cadmium, and lead	ISO 8288
9	Determination of chloride	ISO 9297
10	Determination of sodium and potassium	ISO 9964
11	Determination of *E-coli*	ISO 9308–1

## Data Availability

Data used in this study can be obtained upon request from the corresponding author.

## Appendix

### A. Information on Some Laboratory Tests

#### A.1. General

All the laboratory tests were conducted at the Uganda Industrial Research Institute (UIRI) laboratory. The UIRI laboratory is one of the laboratories in Uganda which is certified by the Uganda National Bureau of Standards. The normative references for the various tests conducted are summarized in Table 4.

#### A.2. Determination of Chemical/Biological Parameters in Water

(i) Chloride was analyzed by placing 20 ml of the sample into a conical flask and 2 to 3 drops of Potassium chlorate (K_2_CrO_4_) added. The mixture was titrated against silver nitrate (AgNO_3_) to a reddish yellow end point (tea color). The concentration of chloride was computed from
  (A.1) $$\begin{array}{c} \text{chloride as Cl},\text{mg}/L=\frac{\text{titrevol of }{\text{AgNO}}_{3}\times \text{normality of }{\text{AgNO}}_{3}\times 35.5\times 1000}{\text{volume of sample taken}}. \end{array}$$
(ii) pH was measured using the multimeter. In the first step, the PH electrode was rinsed with de-ionized water. The multimeter was switched on. The next step was to standardize the multimeter by using buffer solutions of pH 4.01, pH 7.0 and pH 9.2 at 25^o^C. Again, the pH electrode was rinsed with de-ionized water. The next step comprised placing 50 ml of water in a plastic beaker and directly determining pH by immersing the electrode in the water. After two minutes of waiting to ensure the readings stabilize, the pH and temperature were recorded.
(iii) Total dissolved solids (TDS) was also measured using a multimeter. To measure TDS, the steps were as follows:
  (i) Rinse the electrode.
  (ii) Switch on the meter.
  (iii) Place 50 ml of water in a plastic beaker and immerse the electrode.
  (iv) Press the parameter button and select TDS.
  (v) Wait for about 2 minutes for the reading to stabilize and record the TDS reading.
(iv) Sulfates in the water samples was precipitated as Barium Sulfate (BaSO_4_) in the presence of hydrochloric acid (HCl). The precipitate was washed till free from chloride, ignited, and weighed in BaSO_4_. 100 ml of sample was added in a beaker with 2 drops of methyl red indicator. Next, HCl was added drop by drop till the color changed to orange followed by 10 ml of Barium chloride (BaCl_2_) and the mixture was heated to boil for 2 minutes. The mixture was filtered through the Whatman filter paper with addition of hot water until there was no more chloride. The filter paper and its content were transferred into a predried and weighed crucible and ignited in the furnace at 550°C for 2 hours. After 2 hours, the residue was cooled and weighed as BaSO_4_. Sulfate concentration was computed as
  (A.2) $$\begin{array}{c} {\text{SO}}_{4},\text{ mg}/L=\frac{\text{weight of residue }\times 96\times 1000}{\text{Volume of sample}\times 223}. \end{array}$$
(v) Metal ions were determined using the atomic absorption spectrometer (AAS). It involved filtering 30 ml of the sample using a filter paper. Next, the given sample was acidified by adding 2 ml of concentrated nitric acid and readings were taken using AAS. The metal ion concentration was computed from
  (A.3) $$\begin{array}{c} \text{metal ion},\text{mg}/L=\frac{\text{concetration}\left(\text{obtained after reading on AAS}\right)}{\text{volume of sample}}. \end{array}$$
(vi) To determine the nitrates, 1 ml of 5% salicylic acid (HOC6H4CO2H) and sulfuric acid (H_2_SO_4_) were added in 2.5 ml of the sample. 5 ml of 2N solution of sodium hydroxide (NaOH) was added to raise the pH above 12. Absorbance was measured at 410 nm. The concentration of nitrate was calculated as follows:
  (A.4) $$\begin{array}{c} {\text{NO}}_{3},\text{mg}/L=\frac{\text{concetration}\left(\text{obtained after reading on UV}\right)\times \text{dilution factor}}{\text{volume of sample}}. \end{array}$$
(vii) The membrane filtration technique was used for the E-coli test. The sampling bottles were sterilized (by putting them in an oven for 1 hour at a temperature of 160°C) prior to sample collection. The Chromogenic Coliform Agar was used in this test. The powdered agar was first prepared to form a creamy solution that was poured inside Petri dishes and kept in a refrigerator. Clean measuring cylinders were used. A pipette was used to add 0.5 ml of the sample into the cylinders. Next, 99.5 ml of sterile distilled water was then added to obtain 100 ml of the mixture. The 100 ml mixture was added to the disinfected membrane filtration unit using a funnel, the unit turned on to create a vacuum within its core, forcing the water to flow through the filter. The filter paper was put on the agar inside the Petri dishes then covered and inserted in an incubator. The incubator was set at 37°C and the samples were left for 24 hours. After 24 hours, the filter papers were observed for the presence of blue and pink spots on the surface. The pink spots would be a sign of coliforms while the blue spots could indicate the presence of *E. coli*. The value of *E. coli* per sample was obtained using
  (A.5) $$\begin{array}{c} \text{Cfu}/100\text{ml}=\frac{\text{number of colonies}}{\text{volume of sample used}}\times 100. \end{array}$$
